# Worrying About Leadership: Is It a Liability or an Advantage for Leadership of Women and Men?

**DOI:** 10.3389/fpsyg.2022.675522

**Published:** 2022-03-25

**Authors:** Arzu Karakulak, Ayşe Burçin Başkurt, Gamze Koseoglu, Zeynep Aycan

**Affiliations:** ^1^Department of Psychology, Bahçeşehir University, Istanbul, Turkey; ^2^Istanbul Policy Center, Sabanci University, Istanbul, Turkey; ^3^Department of Psychology, Koç University, Istanbul, Turkey; ^4^Department of Management and Marketing, University of Melbourne, Parkville, VIC, Australia

**Keywords:** gender, leadership, stereotype threat, warmth and competence, worries about leadership

## Abstract

Worries about leadership (WAL) is a new construct tapping worries an individual may feel about possible negative consequences of accepting a leadership role. Three studies investigate how WAL is associated with men’s and women’s willingness for leadership and their perceived leadership potential rated by others. The first is a laboratory study on 328 participants, which shows that WAL is negatively associated with women’s willingness for leadership, while it is not related to that of men. The second study, which is a field study with multilevel-nested data from 429 employees and 101 supervisors, reveals that male subordinates are more likely to receive a favorable judgment of leadership potential by their supervisors when their WAL increases, while female subordinates’ WAL is irrelevant to this judgment. The final study, which is an experimental study on 122 supervisors, shows that supervisors view hypothetical male leadership candidates with high WAL as having higher warmth and lower competence (than those with low WAL), which both mediate the effect of WAL on judgments of their leadership potential made by the supervisors. Even though supervisors also view female candidates with high WAL as warmer, this does not evoke higher perceptions of leadership potential. Implications for increasing gender parity in leadership are discussed.

## Introduction

Although women-led organizations are as successful as those led by men (Paustian-Underdahl et al., 2014; Lanaj and Hollenbeck, 2015; Faccio et al., 2016), the gender gap or glass ceiling (Hymowitz and Schellhardt, 1986) prevails in managerial positions (e.g., Lawless and Fox, 2012; Center for American Women and Politics, 2020). Women are still severely underrepresented in high managerial positions, despite their potential for effective leadership. Indeed, only 31 of the Fortune 500 companies are currently led by women CEOs (Catalyst, 2022). Employees, who may be the most suitable for leadership do not always emerge or are selected for this role (Lanaj and Hollenbeck, 2015). Both leadership over emergence (i.e., individuals with little potential to emerge or be selected as leaders) and under emergence (i.e., individuals with high potential to not emerge or not being selected as leaders) may account for women’s underrepresentation in leadership roles; yet extant leadership literature provides insufficient attention to these mechanisms (Hanna et al., 2021). The present research examines the role that worries related to assuming a leadership role may take in the process of leadership under emergence, with particular focus on that of women.

Kossek et al. (2017) reviewed three perspectives on women’s under emergence as leaders and proposed an integrative multilevel model of women’s career equality to lay out “opt-out” and “pushed-out” factors. The three perspectives included in their model are career preferences (i.e., the interaction of women’s interests, values, and goals with work environments and jobs), gender biases and stereotypes (i.e., explicit and implicit gender biases that affect both women’s self-assessments as potential leaders and their perceptions by others), and work-family dynamics (i.e., incompatibility of work and family roles for women). Authors argue that, while studying these perspectives, the literature remains fragmented and fails to integrate the opt-out and pushed-out approaches, which are “…not in conflict but coexist” (Kossek et al., 2017, p. 244).

Traditional leadership research fails to address the opt-out mechanisms and overlooked the role of self-selection mechanisms for leadership (Epitropaki, 2018). Instead, the field has narrowly focused on examining factors that are associated with being perceived as leader-like (Hogan et al., 1994) or examined evaluations about leadership candidates’ potential to emerge as a leader (e.g., Luria and Berson, 2013; Joseph et al., 2015). The individual’s decision to pursue or stay away from leadership roles received little attention (for an exception, see, Chan and Drasgow, 2001). The newly introduced concept of Worries About Leadership (WAL; Aycan and Shelia, 2019) addresses this shortcoming and views leader emergence as an agentic process. WAL is defined as “the worries people have about the possible negative consequences of assuming a leadership role” (Aycan and Shelia, 2019, p. 23). It represents a construct that encounters both leaderships opt-out and pushed-out processes, and maps onto the gender bias and stereotypes perspective proposed by Kossek et al. (2017).

Stereotypes and biases in the domain of leadership favor men and discriminate against women (Schein and Mueller, 1992; Koenig et al., 2011; Powell and Butterfield, 2015). The stereotype content model (Fiske et al., 2002) postulates that stereotypical perceptions of individuals and groups are formed along two universal dimensions, namely warmth (i.e., likability, trustworthiness) and competence (i.e., efficiency, respect) (Fiske et al., 2007). Both leaders and men have traditionally been stereotyped as being high on competence and low on warmth (e.g., Cuddy et al., 2011; Mayseless and Popper, 2019), while women are stereotyped in the opposite way as low on competence and high on warmth (Dardenne et al., 2007). Hence, the stereotypical view of men aligns with that of leaders, while that of women diverges from it (see also Eagly and Karau, 2002).

We assert that leadership stereotypes discriminating against women create a context where the effect of WAL may become more influential on women’s willingness for leadership and their perceived leadership potential whereas stereotypes favoring men may weaken the same for men. We first investigated whether women’s WAL decreases the willingness to accept a leadership role (i.e., opt-out of leadership) more strongly than that of men (Study 1). We further explored whether women’s WAL is more influential than men’s WAL to lower their perceived leadership potential by others (i.e., being pushed-out) (Study 2). Finally, we examined how men’s and women’s WAL reflects differently on their perceived leadership potential *via* gender-stereotypical attributes (i.e., warmth and competence) (Study 3). We tested our hypotheses in three studies using different methodologies, including a laboratory study with a student sample, a field study with a matched sample of supervisors and employees in an organization, and an experimental study with supervisors of the same organization. In all studies, a male-female comparison is drawn to explore the role of gender more comprehensively *vis-à-vis* WAL.

With these studies, we aim to make three contributions: First, we aim to contribute to the burgeoning discussion on self-selection biases (i.e., opt-out processes) in the leader emergence literature (cf., Epitropaki, 2018). There is a growing recognition of the agentic perspectives in leadership research to suggest that not everyone wants to assume a leadership role when the opportunity arises (cf. Chan and Drasgow, 2001; DeRue and Ashford, 2010). Previous research that acknowledged the role of agentic mechanisms mainly studied women’s reluctance for leadership roles as a matter of lacking leadership motivation (Maurya and Agarwal, 2013), having lower career aspirations (e.g., Maurya and Agarwal, 2013; Elprana et al., 2015), and holding weaker desires for attaining powerful leadership positions than men (Gino et al., 2015). Women’s reluctance for leadership may be rooted not only in lack of *wanting* to become a leader but also in perceiving these positions more threatening (Hoyt and Murphy, 2016; Alan et al., 2020). The newly introduced construct of worries about leadership (WAL; Aycan and Shelia, 2019) tackles the perceived threat of holding a leadership position and the associated emotion (i.e., worry) as an obstacle for leadership.

Second, the current study investigates the opt-out and pushed-out processes simultaneously through the lens of WAL. Aycan and Shelia (2019) demonstrated that WAL reduced the likelihood of individuals’ self-nomination for leadership (opt-out) as well as others’ nomination of them for leadership (pushed-out). However, the authors have not explored WAL in relation to gender differences in opt-out and pushed-out processes. In line with the call of Kossek et al. (2017) to study leadership opt-out and push-out processes in an integrated fashion, this paper utilizes WAL and examines how it associates with both willingness for leadership and perceived leadership potential of women and men.

Third, although there have been attempts to investigate the role of emotions in leadership (e.g., emotional contagion between leaders and followers, emotional regulation of leaders; Connelly and Gooty, 2015), we explicitly explored the role of emotions (i.e., worries) to explain the gender divide in the candidacy for leadership. Figure 1 depicts the overview of the three studies reported in this manuscript and how they are integrated.

**FIGURE 1:** Research overview.

## Worries About Leadership

The concept of WAL is grounded in three theoretical perspectives: (1) the anticipation of threatening outcomes creates anxiety (appraisal theory of motivation, Lazarus, 1991), (2) especially when these outcomes pose a threat to the satisfaction of a person’s basic needs (self-determination theory, Deci and Ryan, 1985), (3) resulting in avoidance or withdrawal behavior (self-handicapping theory of regulation, Jones and Berglas, 1978). Anticipated negative consequences of accepting a leadership role may involve failure (i.e., being unsuccessful as a leader), harm (i.e., causing damage to others and oneself), and work-life imbalance (i.e., being unable to meet personal and familial demands) (Aycan and Shelia, 2019). Anticipating failure, harm, and work-life imbalance threatens fulfillment of the need for competence, relatedness, and autonomy, respectively, elevates worries, and results in self-handicapping behavior.

Aycan and Shelia (2019) found empirical support for the WAL construct and its measure based on different study settings and populations. With employee samples in Europe and the United States, WAL was found to tap into a different construct domain than motivation to lead (Chan and Drasgow, 2001) and neuroticism. In the laboratory study of Aycan and Shelia, a lower level of WAL was found to predict self-nomination for the leadership position above and beyond motivation to lead. In their naturalistic field experiment with a longitudinal design, WAL predicted who was elected as a leader by others. Furthermore, in their psychophysiological laboratory study, the correlations between WAL scores and electrodermal and cardiovascular activities were in the expected directions. Thus, WAL may prevent individuals from opting in for leadership and reflect on others by evoking negative impressions regarding leadership potential. In this paper, we extend the research by Aycan and Shelia (2019) and assert that the negative effect of WAL on opt-out and pushed-out processes is moderated by gender.

As stated earlier, implicit and explicit gender stereotypes and biases may create an obstacle for women’s leadership. The reason for this is that leadership stereotypes generally align with the traditional stereotype of men as being high on competence and low on warmth (Cuddy et al., 2011; Mayseless and Popper, 2019) and contrast with the traditional stereotype of women who are typically viewed as being low in competence and high in warmth (Dardenne et al., 2007). On the other hand, the WAL concept seems stereotypically more aligned with women and less with men. The reason is high WAL implies being worried about failing in the leadership role, which is likely to come across as being incompetent. High WAL also implies being worried about harming others and losing work-life balance, which is likely to come across as being warm (e.g., trustworthy, sincere, humane) (Diekman and Eagly, 2008; Cuddy et al., 2011). The divergence in stereotype content between women and leaders likely results in worries related to performing a leadership task being more salient for women compared to men. This aligns with the notion of *stereotype threat* that women experience when facing leadership (Steele, 1997; Spencer et al., 1999). Stereotype threat describes a state of increased physiological stress and self-monitoring that arises when individuals are asked to perform in domains where they expect to be judged or treated according to negative stereotypes (Hoyt and Murphy, 2016). Experience of stereotype threat triggers concerns about performing well (Spencer et al., 1999), leads to stress responses including anxiety (O’Brien and Crandall, 2003), negatively affects performance (Davies et al., 2005; Smith et al., 2015), and promotes withdrawal from tasks and situations associated with the negative stereotype (Elliot and Church, 2003; Schmader et al., 2008). When women are asked to perform a leadership task, the stereotype threat may be activated (Schein et al., 1996), and worries related to leadership may become a stronger barrier for women’s compared to men’s leadership. Eventually, women’s leadership is likely to be guided more strongly by WAL than that of men.

## Study 1: Does Worries About Leadership Operate Differently in Women’s and Men’s Willingness for Leadership?

Biases and negative stereotypes against women as leaders not only affect how others perceive women’s leadership potential but also “lead to self-directed bias in women’s self-evaluation of their fit with male gender-typed jobs (Heilman, 2012) *[*… *and*…*]* shape the development of gender-normative traits (Brown and Diekman, 2010)” (Kossek et al., 2017; p. 234). Women internalize negative stereotypes and regulate their self-perceptions and behaviors accordingly: They feel and perceive themselves as unsuitable for leadership, which makes them eventually withdraw from tasks and activities associated with leadership (see Wood and Eagly, 2002; Kossek et al., 2017). There is evidence showing that biases and negative expectations may drain women’s aspirations for managerial positions (Coffman and Neuenfeldt, 2014) and make them adopt a strategy of “intentional invisibility” (Ballakrishnen et al., 2018, p. 24) so that they become more likely to opt themselves out of leadership. In a situation where the opportunity for leadership arises, women are likely to experience stereotype threat, which promotes a mental state where decisions and behaviors are more strongly guided by fears and worries (Spencer et al., 1999; Elliot and Church, 2003; O’Brien and Crandall, 2003; Schmader et al., 2008). Hence, women’s WAL will likely become more influential on their willingness for leadership than that of men who will find themselves in a situation that is compatible with their gender stereotype, and thus not threatening.

### Hypothesis 1

Gender will moderate the negative effect of WAL on the willingness for leadership in such a way that this relationship is stronger for women than it is for men.

### Study 1 Method

#### Participants and Procedure

We recruited voluntary student participants through the subject pool of a private university located in Turkey^1^. The participants who completed the two-part group decision-making experiment received course credit. The study featured a betting game adapted from an experiment of behavioral economics (Ertac and Gurdal, 2012), in which teams earned $0 to $25 and then divided the winnings evenly among the five team members. In the first part of the study, the participants reported their level of WAL *via* an online survey. After 1 to 3 weeks, the participants came to the laboratory to complete a group decision-making task involving financial risk for the participants. When the participants arrived at the laboratory, they were randomly assigned to groups of five. We ensured that the five group members were strangers. The experimenter explained the procedures and then sent each group to another room where they were seated in circles and asked to *not* interact. Each participant was required to make a private money allocation decision on behalf of his or her group. A group budget of $10 had to be divided between a safe and risky option. The amount put into the safe option would be maintained, but the money earned from the risky option would be multiplied by the factor 2.5 or entirely lost, depending on the outcome of the coin tossing. Hence, each group could earn between $0 and $25. After the participants made their allocation decisions, they were asked to indicate their willingness to be their group’s final decision makers, which served as the dependent variable of this study. The participants were informed that the allocation decision of only *one* group member would be implemented. The name of the decision-maker was randomly drawn among all the members who answered affirmatively to becoming the group’s leader, or among all the five group members if all answered negatively. We had assessed WAL before the decision-making sessions to avoid priming effects. We merged data from both parts of the study according to individual codes that each participant generated at the beginning of both sessions.

The final sample included 328 undergraduate students enrolled in an introductory psychology course (59% women, *M*_*age*_ = 19.8 years), forming in total 71 groups^2^. Data were collected across four semesters.

### Measures

#### Participant Gender

The participants indicated their gender (i.e., biologically determined sex) on a paper and pencil questionnaire, which we used to identify participant gender (0 = man; 1 = woman).

#### Worries About Leadership

We used the 16-item measure developed by Aycan and Shelia (2019). We asked the participants to imagine that they were offered a leadership role in one of the major student clubs and to indicate the extent of their worries about “being exposed to more criticism,” or “losing self-esteem in case of failure” (i.e., worries about failure); “being unable to balance work and family,” or “having less time for myself (e.g., hobbies)” (i.e., worries about work-life imbalance); and “hurting others’ feelings in the work context by the decisions I make,” or “treating employees unfairly” (i.e., worries about harm) on a 5-point Likert-type scale from 1 = *to a very little extent* to 5 = *to a very large extent.* Cronbach’s α internal consistency was 0.85.

#### Willingness for Leadership

To measure this construct, we adopted the measure of Ertac and Gurdal (2012) and asked the respondents to report their willingness to be the decision-makers for their groups, on a 5-point Likert-type scale from 1 = *not at all* to 5 = *very much*^3^.

### Study 1 Results

Table 1 shows descriptive statistics and correlations of the study variables for the total sample, men and women. To test whether the prediction effect of WAL differs by gender, a moderation analysis using Model 1 of the Hayes (2012) PROCESS macro with a bootstrapping procedure of 5,000 resamples was performed. The centered score of WAL was entered as a predictor, and the gender was entered as a moderator to predict the willingness for leadership. Our analysis revealed that the regression model was significant [*R*^2^ = *0.09, F_*change*_* (3, 320) = 10.83, *p* < 0.001]. In this model, willingness for leadership was significantly predicted by gender (β = −*0.42*, *t*(323) = −4.82, *p* < 0.001), and by the interaction between gender and WAL (β = −*0.31*, *t*(323) = −2.06, *p* < 0.05) (see Table 2). Exploration of WAL’s prediction effect by gender revealed that WAL did not predict men’s willingness for leadership [β = 0.07, *t*(127) = 0.53, *p* = 0.60), but it negatively predicted women’s willingness for leadership (β = −*0.25*, *t*(195) = −2.88, *p* < 0.01; Figure 2], providing support to Hypothesis 1.

**TABLE 1:** Study 1 descriptive statistics and correlations.

Total Sample (*N* = 328)	Mean	*SD*	1	2	3
1 Participant’s Gender	0.61	*0.49*	1	−0.23***	0.07
2 Willingness for Leadership	3.58	*0.80*		1	-0.15**
3 WAL	3.12	*0.61*			1
Women (*N* = 198)	Mean	*SD*	1	2	3
2 Willingness for Leadership	3.41	*0.80*	−	1	−0.20**
3 WAL	3.16	*0.64*	−		1
Men (*N* = 129)	Mean	*SD*	1	2	3
2 Willingness for Leadership	3.84	*0.74*	−	1	0.05
3 WAL	3.06	*0.55*	−		1

**p < 0.01, ***p < 0.001, gender coded as 0 = men, 1 = women.

**TABLE 2:** Study 1 regression results.

	Unstandardized beta (*SE*)	*t*	*p*	LLCI	ULCI
Constant	3.84 (*0.87*)	55.99	0.000	3.71	3.98
Participant’s Gender	−0.42 (*0.88*)	−4.82	0.000	−0.60	−0.25
WAL	0.07 (*0.13*)	0.53	0.594	−0.18	0.32
Participant’s Gender × WAL	−0.31 (*0.15*)	−2.06	0.040	−0.61	−0.01

*Gender coded as 0 = men, 1 = women.*

**FIGURE 2:** Worries about leadership’s effect to predict women’s and men’s willingness for leadership in Study 1.

### Study 1 Discussion

The first study was a laboratory study examining whether WAL had a stronger negative effect on women than men to predict willingness for leadership. Our analyses revealed that the effect of WAL operated differently on women’s and men’s willingness for leadership. WAL had a negative effect for women but not for men in reducing the willingness for leadership, as predicted by Hypothesis 1. As such, women who reported higher WAL were more likely to opt themselves out of leadership than women with low WAL, while men’s WAL was found unrelated to their willingness for leadership. One possible explanation for the absence of WAL’s effect on men’s willingness for leadership could be that the task of making a risky decision on behalf of a group may have been too weak to evoke men’s worries about leading the group. Such decisions (i.e., those involving risk and money) may be perceived as naturally falling in the domain of responsibility for males (Byrnes et al., 1999). Therefore, the WAL level may be irrelevant when volunteering for a task seen almost like a natural duty for males. In contrast, the task was sufficient to evoke women’s worry and to impair their willingness for leadership. Making a risky decision involving money on behalf of the group is likely to induce stereotype threat for women (Hoyt and Murphy, 2016) so that WAL becomes a self-set barrier. It should be noted that gender moderated WAL’s effect despite equal levels of self-reported WAL among men and women. While we did not hypothesize for any gender differences in regard to the level of WAL, we acknowledge that the absence of such gender difference may also be related to our study design, and caused by the fact that WAL was assessed independent from and prior to the leadership task. It is thus likely that the level of self-reported WAL of women would have been higher than that of men, if WAL was assessed right at the leadership situation.

Overall, results obtained from the first study support the notion that bias and stereotypes in the leadership domain affect women’s self-evaluation as leaders *via* the experience of WAL (Kossek et al., 2017). While men with high WAL did not abstain from assuming leadership, women with high WAL preferred to opt themselves out of leadership. Due to the laboratory nature of the study, our sample consisted of university students, and leadership had to be limited to one of the key tasks of leadership, namely, making a risky decision that impacts the group members (Yukl, 2012; Ertac et al., 2020). While this may be seen as limiting the external validity of the present research, the fact that our findings align with previous laboratory studies finding that women reported less willingness for leadership than men (e.g., Ertac and Gurdal, 2012; Ho et al., 2012; Lanaj and Hollenbeck, 2015; Born et al., 2020; Ertac et al., 2020) strengthens the validity of the present results. Moreover, evidence from meta-analytical reviews suggests that differences between student and non-student samples in regard to organizational research findings seem rather minimal (Wheeler et al., 2014, p. 10). In addition, even though it may seem that leadership is a topic of little concern to university students, research shows that leadership roles beyond the occupational domain (e.g., in family, schools or extracurricular activities) seem to predict leadership in the professional domain (Arvey et al., 2007), suggesting that WAL may well be relevant for students too. By using the same research paradigm, Alan et al. (2020) found that, while there were no gender differences in willingness for leadership among children, with entering adolescence the proportion of girls who volunteer for leadership dropped by 39%, suggesting that processes of opting out from leadership may start from adolescence. Still, further research that moves beyond a laboratory setting and utilizes samples other than university students, as we conducted in our second study, seems advisable to further test the robustness of the present results.

## Study 2: Does Worries About Leadership Make a Difference in How Others Perceive Men’s and Women’s Leadership Potential?

In line with Kossek et al. (2017) conceptualization of leadership to encounter both opt-out and pushed-out processes, Study 2 shifts the focus away from the role of WAL in opting out of the leadership to its role in being pushed out of the leadership domain, operationalized as supervisors’ judgment of leadership potential (cf., Luria and Berson, 2013).

Aycan and Shelia (2019) argued that WAL may inform others about leadership potential *via* two channels. First, high WAL may be sensed by others through embodied worries (Melina et al., 2013). For instance, those with salient worries may experience higher physiological arousal while discussing the possibility of becoming a leader, shown as nervousness in speaking, increased sweating, increased respiratory activity, shaky hands, and a flushing face (Boiten et al., 1994; Cacioppo et al., 2000). Second, high WAL may provoke self-handicapping behavior, making people less likely to appear on the radar searching candidates for leadership. Those with higher worries would withdraw from leadership-related activities (e.g., trainings, self-promoting activities), signaling a lack of interest and low potential for leadership to others.

Such WAL-reflective physiological reactions and withdrawal behaviors are likely to be interpreted differently for men and women. Evidence shows that, even if men and women show the same behavior at work, they are still perceived and treated differently (e.g., Rudman and Glick, 1999; Turban et al., 2017); namely in a way that is affected by gender stereotypes. Thus, we argue that women with high WAL would experience a double bind (due to their gender and WAL levels) and be pushed out of leadership (i.e., receive the least favorable judgment of leadership potential) more strongly than men with high WAL. When women’s WAL is sensed by others, the stereotypical perception that women lack leadership potential may be further strengthened. However, when men’s WAL is sensed by others, stereotypes favoring men for leadership (Powell and Butterfield, 2015) may buffer against the negative effect of WAL on perceived leadership potential. Consequently, we argue that women’s WAL will play a more detrimental role for their perceived leadership potential than men’s WAL.

### Hypothesis 2

Gender will moderate the negative effect of WAL on perceived leadership potential in such a way that this relationship is stronger for women than it is for men.

### Study 2 Method

To test our hypothesis, we collected multilevel nested data from 429 employees and their 101 department supervisors working for 23 different shops of a retail company located in Turkey, producing textile goods^1^. The response rate for employees was 35%; the response rate for supervisors was 62%. Employees averaged 25.4 years old and 3 years in the organization; 62.4% were women. Department supervisors averaged 29 years old and 6.36 years in the organization; 64.7% were men. The multisource nature of our data reduced risks of common method bias (Podsakoff et al., 2003). The employees provided self-reported data on WAL and gender; the supervisors reported ratings of leadership potential for each employee who responded to the WAL survey. All data were collected *via* paper-and-pen surveys.

### Measures

#### Worries About Leadership

We used the same 16-item WAL scale (Aycan and Shelia, 2019) used in Study 1. Cronbach’s alpha for this sample was 0.90.

#### Gender

Employees reported their gender (i.e., biologically determined sex) in the employee survey (0 = woman; 1 = man). To control for the effect of departmental supervisors’ gender, the supervisors were also asked to indicate their gender in the supervisor survey.

#### Perceived Leadership Potential

The supervisors had an average of four subordinates. Adopting the approach of General Leadership Index (Lord et al., 1984), we asked the supervisors to evaluate each subordinate’s leadership potential after rating them on several performance indicators using a single item: “I believe this employee has what it takes to be promoted” *1* = *strongly disagree* to *5* = *strongly agree*. In the organizational context of this study, promotion implied a mid-level managerial position in which leadership responsibilities involved managing teams and giving strategic and operational decisions in a semi-autonomous way.

### Study 2 Results

The department supervisors rated their employees nested within their departments. To analyze this data set, we used HLM 7.02 to test our nested data and hypothesis (Raudenbush et al., 2011). To evaluate the multilevel data, we first ran a null model with perceived leadership potential as the only criterion variable, without predictors (Hofmann et al., 2000). According to this model, the ICC (1) for the criterion variable was 0.16, suggesting that 16% of the variance of this variable existed between the department supervisors who rated their employees. Therefore, it was appropriate to take a multilevel approach to take the between-level variance into account. We performed a hierarchical multilevel linear regression model with employee gender, WAL, and their interaction to predict perceived leadership potential. We lacked a theoretical rationale to expect that slopes would vary among departments. Because of the low between-group variance for WAL [i.e., ICC (1) = 0.002], our model did not specify random slopes. In addition, we compared the deviance scores (calculated as -2*loglikelihood) of the random coefficient and random slopes models to see whether the data fit with one or the other significantly better than the other (Campbell and Kashy, 2002). The deviance score of the random coefficient model was 1230.50. The deviance score of the random slopes model was smaller (deviance = 1219.25). However, the chi-square test suggests that the difference between the deviance of the random slopes model and the random coefficients model was not significant [χ^2^ (9, *N* = 428) = 11.25, *p* > 0.05], indicating that the random slopes model was not statistically better than the random coefficients model. As the models were not statistically different, for the sake of parsimony, and considering the low between-group variance for WAL, we decided that continuing with the random coefficients model was more appropriate (Snijders and Bosker, 1999). As grand-mean centering creates inappropriate Level-1 estimators by generating regression slopes that are a mixture of within and between variations (Raudenbush and Bryk, 2002; Enders and Tofighi, 2007), Level-1 variables were group mean centered. Table 3 shows descriptive statistics and correlations. As Table 4 shows, we found a significant interaction effect (γ = 0.40, *p* < 0.01) between the employees’ gender and their WAL to predict their leadership potential rated by their supervisors, whereas employees’ WAL had a marginally significant negative effect (γ = −0.14, *p* = 0.09), and their gender (0 = woman, 1 = man) had a positive and significant main effect (γ = 0.32, *p* < 0.01). Specifically, Figure 3 shows that WAL had a positive and significant relationship with perceived leadership potential for men (γ = 0.31, *p* < 0.05). For women, the relationship was negative but non-significant (γ = −0.14, *p* = 0.098). Therefore, our findings did not support Hypothesis 2.

**TABLE 3:** Study 2 descriptive statistics and correlations.

	Mean	*SD*	1	2	3	4
1 Perceived Leadership Potential	3.16	*1.04*	1			
2 Candidate’s WAL	3.52	*0.83*	−0.03	1		
3 Candidate’s Gender	0.38	*0.49*	0.13**	−0.08	1	
4 Supervisor’s Gender	0.64	*0.48*	−0.02	−0.01	0.17**	1

N = 428, **p < 0.01, gender coded as 0 = women, 1 = men.

**TABLE 4:** Study 2 multilevel regression results.

	Model 1	Model 2	Model 3
**Level 2 Controls**			
Supervisor’s Gender	−0.02 (0.13)	−0.02 (0.13)	−0.02 (0.13)
**Level 1 Independent Variables**			
Employee’s WAL		−0.001 (0.07)	−0.14 (0.08)^†^
Employee’s Gender		0.32 (0.13)	0.32 (0.12)**
**Interaction Variables**			
Employee’s WAL × Employee’s Gender			0.40 (0.14)**
Deviance	1238.92	1237.92	1230.50

γ values and standard errors are reported for N (individuals/employees) = 429, N (departments/supervisors) = 101; gender coded as 0 = woman, 1 = men; **p < 0.01; ^†^p < 0.10; deviance is calculated as −2 * loglikelihood.

**FIGURE 3:** Interaction effect between WAL and gender on perceived leadership potential in Study 2.

### Study 2 Discussion

Our analysis showed that gender moderated WAL’s effect on perceived leadership potential but in a different way than what we hypothesized. Specifically, although WAL had a non-significant effect on the perceived leadership potential for women, it positively affected that of men. Taken together, our results obtained from the first two studies indicate that WAL plays out differently for leadership candidacy of men and women: WAL was positively related to men’s leadership potential rated by their supervisors and was not related to their willingness for leadership, whereas WAL was unrelated to women’s leadership potential rated by their supervisors and negatively related to their willingness for leadership. The absence of a WAL effect for women, together with the main effect of a candidate’s gender, suggests that women’s leadership potential seems to be evaluated independently from their WAL levels and their leadership qualities but based on their gender only. For men, on the other hand, perceptions of their leadership seem to be associated both with the stereotypical perception that men are naturally competent leaders (Cuddy et al., 2011; Katila and Eriksson, 2013), and their personal leadership qualities. Men were generally rated as having higher leadership potential than women, and men with high WAL were rated more favorable in terms of leadership potential than those with low WAL.

The asymmetry between WAL’s effect on men’s versus women’s leadership potential suggests that WAL may not directly but rather indirectly influences the perception of leadership potential. A first explanation may be that WAL manifests itself differently for men versus women. The same level of WAL may transform into different behaviors (i.e., embodied worries, withdrawal behaviors) among men versus women, and thereby differently affect the perception of leadership potential. High WAL in men may be externalized in a different way than high WAL in women so that the behaviors men show would not reflect that they are worried. Additionally, men with high WAL may exhibit higher levels of performance and devote more effort in self-promoting behaviors as they do not consider WAL as a barrier to leadership, while women with high WAL would perform self-handicapping behaviors. Supervisors that judge leadership potential of their subordinates may base their evaluations on such observable reflections of WAL (Aycan and Shelia, 2019). This argument aligns with previous research, which showed that people seem to perceive others more strongly on the basis of external inputs, such as their observable behaviors and actions, while self-perception is more strongly tied to internal inputs such as emotions and feelings (Pronin et al., 2001; Pronin, 2008).

Yet, a second explanation could be that men’s versus women’s expressions of WAL may be perceived differently despite the equally reflected worries, namely in a way governed by gender stereotypes. As stated, there is evidence showing that women and men are treated differently at work despite showing the same behaviors and communication patterns at work (e.g., Turban et al., 2017).

Building on the stereotypes and bias perspective that is put forward by Kossek et al. (2017), we draw on the second interpretation explained above and assert that WAL could transform into judgment of leadership potential of men versus women (despite equal expressions of WAL) *via* stereotypes. A good way of testing this claim would be to assess the WAL of employees and to contrast that with the assessments of WAL made by the supervisors. Another possibility for testing this claim would be to make the WAL levels of male and female leadership candidates explicitly visible to those who judge leadership potential and to examine how low versus high levels of WAL is stereotypically perceived, and how these perceptions transform into ratings of perceived leadership potential of men versus women. We adopted the latter strategy in our third study. The third study aims at resolving the seemingly paradoxical (i.e., positive) effect of men’s WAL on their perceived leadership potential through an experimental study where WAL and gender are manipulated, and perceptions of warmth, competence, and perceived leadership potential are assessed.

## Study 3: Do Perceptions of Warmth and Competence Mediate the Link Between Worries About Leadership and Perceived Leadership Potential of Women and Men?

Social perception research suggests that the two dimensions of the stereotype content model, warmth, and competence account for more than 80% of the variance in perception of groups and individuals, as well as abstract categories such as leaders (Fiske et al., 2007). Warmth and competence underlie impression formation and represent fundamental attributes for mapping stereotypical perceptions. It is possible that individuals’ WAL may also affect the extent to which they are perceived to be warm and competent.

People who have high WAL tend to worry that leadership demands may cause them to harm others, to damage work-life balance, and to fail as leaders (Aycan and Shelia, 2019). Such worries may be associated with good naturedness, sincerity, humaneness, the qualities that signal warmth (Fiske et al., 2007; Cuddy et al., 2011). High WAL people may signal concern for employees (i.e., harming subordinates *via* critical decisions such as discharge), concern for social relationships (i.e., hurting others in close relationships by not being able to balance work and life), and concern for the organization (harming the organizational bottom line due to poor performance in leadership). Indeed, research has confirmed that individuals who reject causing harm to others are judged as more trustworthy (i.e., warm) (Everett et al., 2016). Yet, these worries may also imply a lack of aptitude or confidence to handle these challenges, and thus may be inversely associated with confidence, competitiveness, and intelligence - qualities that reflect competence (Fiske et al., 2007; Cuddy et al., 2011). Thus, high WAL likely suggests being viewed incompetent but warm, which converges with the stereotypical perception of women (Rudman and Glick, 1999; Williams et al., 1999) and diverges from the stereotypical perception of men. As such, we first predicted that high WAL is associated with the perception of high warmth and low competence.

### Hypothesis 3

Higher WAL will lead to higher perceptions of warmth and lower perceptions of competence.

Stereotypical perceptions of warmth and competence are likely to be associated with the judgment of leadership potential. Even though leaders have traditionally been stereotyped as being high on competence and low on warmth (e.g., Cuddy et al., 2011; Mayseless and Popper, 2019), research found that both warmth (also known as communion) and competence (also known as agency) were instrumental to judging leadership potential and effectiveness (Dardenne et al., 2007; Cuddy et al., 2011). Warmth is an attribute that is required and desired in today’s leadership environment. For instance, the recent research by Laustsen and Bor (2017) found that warmth was more influential than competence for the evaluation of political candidates. Bor (2020) found that both warmth and competence serve as mediators between economic perceptions and voting for a political leader. As such, we propose that WAL may indirectly reflect on perceptions of leadership potential *via* the two core dimensions of social perception, warmth, and competence. We expect perceptions of warmth and competence to mediate the relationship between WAL and perceived leadership potential: Higher WAL increases perceptions of warmth and decreases perceptions of competence (as per Hypothesis 3), which is, in turn, positively associated with judgment of leadership potential.

We further expect that, due to prevailing gender biases (Kossek et al., 2017) the way WAL transforms into perceptions of warmth and competence, and how these eventually affect perceived leadership potential may be moderated by gender. Expectation violation theory (EVT; Jussim et al., 1987) posits that individuals judge others more strongly based on behaviors that violate rather than confirm stereotypes. The perception of high warmth and low competence (evoked by high WAL) may be perceived as an expectation violation for men. As such, we propose that the WAL manipulation will have a stronger effect on men’s as opposed to women’s perceived leadership potential.

### Hypothesis 4

Gender will moderate the indirect relationship between WAL and perceived leadership potential through perceptions of warmth and competence, such that this relationship would be stronger for men than for women.

### Study 3 Method

#### Participants

Different organizational settings may evoke varying evaluations and perceptions of leadership qualities (Eagly and Karau, 2002), so, for Study 3, we held the organizational setting constant by recruiting the same supervisors recruited in Study 2. We re-contacted 122 supervisors (*M*_*age*_ = 31.2, 73% men) to answer a brief online questionnaire about their impressions regarding fictitious cases of candidates for a leadership position (response rate, 75%). Seventeen supervisors were excluded for failing to answer our attention check question correctly. We ended up with a final sample of 105 supervisors (*M*_*age*_ = 31.2, 72% men).

#### Procedure and Experimental Manipulation

We used a 2− × −2 between-subjects experimental design, with gender (male vs. female) and a WAL level (low vs. high) of a fictitious candidate for a leadership position as independent variables. The supervisors were randomly assigned to view one of the four profiles of a candidate with a common male or female name, identified as having low or high WAL. More specifically, the supervisors were asked to judge this candidate’s leadership potential based on the candidate’s WAL profile presented to them. The profile included a subset of the WAL measure used in Studies 2 and 3. We selected four of the original 16 items representing worries about failure, work-life imbalance, and harm. The supervisors assigned to the low WAL condition viewed a profile in which the candidate ostensibly gave low scores to these items (either 1 or 2 out of a 5-point scale). The supervisors assigned to the high WAL condition viewed a profile in which the candidate gave high scores to the same WAL items (either 4 or 5 out of a 5-point scale). The supervisors were told that the candidate had consistently high job performance. We added this information to prevent the supervisors from being affected by stereotypical, often implicit, beliefs about job performance according to gender. The supervisors indicated their perceptions of the warmth and competence of the candidate and rated the candidate’s leadership potential for the same type of position used in Study 2.

### Measures

#### Manipulation Check

We asked the participants to indicate how much they agreed that the candidate whose profile (i.e., responses to WAL item) they had seen was worried on a 5-point scale ranging from *1* = *totally disagree* to *5* = *totally agree*.

#### Warmth and Competence

To assess perceptions of warmth and competence, we used the 9-item measure by Fiske et al. (2002), which assesses warmth by asking the participants to rate whether they perceive subjects as *tolerant, warm, good-natured*, and *sincere*, and competence by asking whether they perceive subjects as *competent, confident, independent, competitive*, *and intelligent.* Answer options ranged from *1* = *totally disagree* to *5* = *totally agree*. The mean score obtained from the four items was the measure of warmth; the mean score obtained from the five items was the measure of competence; higher scores indicated higher warmth and competence. Cronbach’s alpha for internal consistency was 0.78 for warmth and 0.74 for competence.

#### Perceived Leadership Potential

Leadership potential of the fictitious candidate was evaluated by the same item used in Study 2 (“I believe this employee has what it takes to be promoted in my store”) with answer options ranging from *1* = *strongly disagree* to *5* = *strongly agree.*

### Study 3 Results

We first checked whether our manipulation of WAL evoked the respondents’ perceptions of worries about the leadership of the fictitious candidate. Results of the univariate ANCOVA with candidate gender and WAL condition as independent variables, the respondent’s gender as a covariate, and perceptions of being worried as the dependent variable confirmed the intended effect [*F*(1,100) = 24.76, *p* < 0.001, partial η^2^ = 0.20]. The respondents in the low WAL condition rated the candidate as less worried (*M* = 2.91, *SD* = 1.26, *SE* = 0.17) than the respondents in the high WAL condition (*M* = 4.04, *SD* = 1.10, *SE* = 0.15), regardless of the gender manipulation.

To examine whether the WAL level influenced the perception of warmth and competence (Hypothesis 3), we carried out an independent samples *t*-test with the WAL level as independent variable and warmth and competence ratings as dependent variables. Descriptive statistics and correlations are presented in Table 5. Our analyses showed that the manipulation of WAL significantly affected perceptions of the candidates’ warmth, *t*(103) = −2.70, *p* < 0.01, Cohen’s *d* = 0.53 but remained irrelevant for ratings of competence, *t*(103) = 0.48, *p* = 0.63.

**TABLE 5:** Study 3 descriptive statistics and correlations.

		WAL	Warmth	Competence	PLP
Male Candidate *n* = 54	M (*SD*)	−	3.56 (*0.67*)	3.28 (*0.84*)	3.02 (*0.96*)

	(1)	1	0.29*	−0.27^†^	−0.25^†^
	(2)		1	0.21	0.32*
	(3)			1	0.69***
	(4)				1
Female Candidate *n* = 51	M (*SD*)	−	3.41 (*0.69*)	3.26 (*0.75*)	3.04 (*1.10*)
	(1)	1	0.23	0.21	0.22
	(2)		1	0.24^†^	0.42**
	(3)			1	0.46**
	(4)				1

WAL = worries about leadership; PLP = perceived leadership potential; *p < 0.05; **p < 0.01; ***p < 0.001; ^†^p < 0.10.

To test whether perceptions of warmth and competence had different mediating effects on the relationship between WAL and perceived leadership potential of male versus female candidates, we performed multi-group structural equation modeling using AMOS. We tested whether a mediation model that linked the WAL manipulation to ratings of perceived leadership potential *via* perceptions of warmth and competence was operating differently for the male versus the female candidate. Additionally, we controlled for possible effects of the supervisor’s gender on ratings of perceived leadership potential (see Figure 4). Results revealed an excellent model fit for the unconstrained model with χ^2^ (4, *N* = 105) = 3.91, *p* = 0.418, RMSEA = 0.00, CFI = 1.00, while the structural weights solution was fitting the data significantly worse (CFI = 0.93, ΔCFI = 0.07). Hence, while the structure of the model seemed to be appropriate to describe the indirect relations between WAL and perceived leadership potential, the strength and/or directions of these relationships were significantly different for the male versus the female candidate. Examination of the standardized regression weights per candidate gender group under the unconstrained model suggests that, while both the perceptions of warmth and competence were conducive for judging men’s and women’s leadership potential (i.e., they both positively related to ratings of leadership potential), the WAL manipulation for the female candidate did not inform the respondents about their warmth and competence. For the male candidate, the high WAL manipulation both decreased the competency ratings and increased the warmth ratings of the candidate, which confirms Hypothesis 4 (Figure 4).

**FIGURE 4:** Results of the multi-group SEM mediation model in Study 3. The first regression coefficient represents the standardized regression weight under the unconstrained model for the female candidate; the second coefficient represents the same for the male candidate; error terms of warmth and competence were correlated; *p < 0.05, **p < 0.01, ***p < 0.001, ^†^*p* < 0.10.

### Study 3 Discussion

The goal of the third study was to examine how high and low levels of WAL are stereotypically perceived along the two universal dimensions of social perception, warmth, and competence (Fiske et al., 2002) and to test whether these perceptions exert a mediator effect between WAL and perceived leadership potential for the male and the female leader candidates. Moreover, we were interested in examining whether potential mediating effects *via* warmth and competence were different for the male versus the female candidate. Specifically, Study 3 was also conducted to shed light on the seemingly paradoxical positive effect of high WAL on men’s perceived leadership potential. The experimental investigation revealed that the WAL manipulation affected ratings of warmth in the hypothesized direction, while it seemed unrelated to the rating of the candidates’ competence. However, results obtained by the moderated mediation analysis revealed the WAL manipulation operated differently for male and female candidates. We found that high WAL increased warmth perceptions and decreased competence perceptions of the male candidate, but not the female candidate (Figure 4). While such a result partly confirms the third hypothesis, stating that higher WAL is associated with higher perceptions of warmth and lower perceptions of competence, it also aligns with the premises of EVT (Jussim et al., 1987). Men who have high WAL would violate gender expectations and thus appear especially high in warmth and low in competence. Women with high WAL, however, seem to be evaluated no differently than women with low WAL. As, in Study 2, women’s WAL turned out to be irrelevant for how they are perceived from outside, which implies that gender stereotypes are more prevalent than women’s personal attributes for judging women as warm and competent in the work context.

Drawing on EVT, we further tested whether the role of warmth and competence as potential mediators between WAL and perceived leadership potential is moderated by the candidate’s gender. Our moderated mediation analysis revealed that high WAL decreased the perception of leadership potential *via* lower ratings of competence for the male candidate, but not for the female candidate. We further found that high WAL also increased the perception of leadership potential *via* higher ratings of warmth for the male candidate, but not for the female candidate, which confirms Hypothesis 4. Overall, our results suggest that high WAL of females had no implications for judging their warmth, competence, and thus their leadership potential. While this result signals that women with high WAL are not perceived as less suitable for leadership, it also signals that those with low WAL women do not receive a leadership advantage. Even though the female candidate’s evaluation as warm and competent was positively associated with their perceived leadership potential, their WAL did not function as a cue to inform others about their warmth and competence. Overall, and together with the results obtained in the second study, our findings seem to be indicative of overreliance on gender stereotypes when judging women’s leadership potential. It seems that biased and stereotypical perceptions dominate over the effect of WAL, and push women out from leadership positions regardless of their personal attributes.

For the male candidate, however, our analyses confirmed an indirect effect of WAL on perceived leadership potential through competence and warmth. Overall, our findings indicate that male candidates with higher WAL are perceived as less competent than males with lower WAL, which then negatively relates to their ratings of leadership potential. However, males with higher WAL are also perceived as having higher warmth than males with lower WAL, which then positively relates to ratings of leadership potential (Figure 4). As such, the effect of WAL on men’s leadership potential perceived by others appears to be ambivalent.

When comparing the results obtained for the males in the second study with the results of the present study, differences in the association between WAL and perceived leadership potential become evident. While the direction of this association was positive in Study 2, the association between WAL and perceived leadership potential was negative by tendency (as not significant) in Study 3 (see Table 5). As already noted, Study 3 employed an explicit manipulation of employees’ WAL where the WAL scores of the candidates were directly visible to the supervisors, while, in Study 2, the supervisors were not informed about the WAL level of their subordinates, and judged their perceived leadership potential on the basis of subordinates’ observable behaviors and actions at work. This implies that WAL may affect the perception of men’s perceived leadership potential through two interconnected paths. On the one hand, males may externalize their WAL differently so that the behaviors of men with high WAL do not signal high levels of worry, and are not perceived by their supervisors as worry. On the other hand, the results of the present study suggest that, even if supervisors accurately perceive men’s WAL, they may still gain leadership advantage through enhanced perceptions of warmth.

## General Discussion

Drawing on the gender bias and stereotypes perspective proposed by Kossek et al. (2017), our objective was to examine whether leadership-related worries (WAL) may provide an additional explanation for why women (and men) opt out and are pushed out of leadership. In Study 1, we examined whether WAL was associated with men’s and women’s willingness for leadership in a group-decision making task involving financial risk. As hypothesized (Hypothesis 1), WAL operated differently on women and men; while women with high WAL were more likely to opt themselves out of leadership, men with high WAL did not abstain from leadership. As such, our results imply that WAL is part of self-selection bias in leader emergence for women, but not for men (Epitropaki, 2018).

In Studies 2 and 3 where we focused on WAL’s effect on pushing out men and women from leadership, we found further support for the gender-divergent effect of WAL; in Study 2, WAL was positively related to ratings men receive for their leadership potential while it was unrelated to those women received. In Study 3, where WAL levels were made visible to the supervisors, perceptions of warmth and competence mediated the relationship between WAL and perceived leadership potential for men but not for women. These findings in combination suggest that high WAL in men may create an advantage for men’s perceived potential for leadership. Aligned with EVT (Jussim et al., 1987), in Study 3, the supervisors viewed high WAL as conveying positive signals about men’s warmth, which, in turn, lead to higher ratings of men’s leadership potential. However, high WAL in men was not entirely positive but signaled ambivalent qualities concerning leadership potential, while explicit WAL was found conducive for men’s perceived leadership potential *via* enhanced perceptions of warmth. Indeed, recent evidence has suggested that perceptions of warmth seem to become increasingly important for leader perception (Laustsen and Bor, 2017; Bor, 2020; Vroman and Danko, 2020). Thus, perceptions of warmth can be an important mechanism causing the seemingly paradoxical positive effect of WAL to predict the perceived leadership potential of men in the second study. However, in Study 3, we also found that high WAL decreased the perceived leadership potential of male candidates *via* decreased perceptions of competence. This, on the other hand, implies that the male employees with high WAL in Study 2 were not perceived by their supervisors as worried, and that the male employees possibly did not perform behaviors that would make them look worried. Instead, the high WAL men in Study 2 may have engaged in self-promoting behaviors that had signaled their interest in leadership. As such, our results suggest that the WAL of men and women may not only reflect differently on others *via* different types of behaviors that benefit men’s perceived leadership potential but is also judged differently when WAL is made visible. Even when men and women are rated as similarly worried (as it was the case in Study 3), men may still gain a leadership advantage through enhanced perceptions of warmth.

For women, on the other hand, findings from both Studies 2 and 3 suggest that their WAL is not influential on their perceived leadership potential. An intriguing question to be explored in future research is why low WAL did not benefit women. It may be due to the backlash effects (Rudman and Glick, 2001). For instance, women with low WAL may be considered assertive and dominant, which creates a “double bind” for them (Eagly et al., 2007). Biased and gender-stereotypical perceptions against women as leaders seem to prevail in creating diverging effects of WAL found in the present research. The negative gender biases against women as leaders may have overridden the effect of WAL and perpetuated the perception that women lack leadership potential (Schein et al., 1996). This interpretation aligns with the biases and stereotypes perspective proposed by Kossek et al. (2017) and converges with the findings of the current research.

## Theoretical and Practical Implications

The present research extends existing leadership literature in several ways. First, our findings contribute to the literature on women’s underrepresentation in leadership. By using the novel construct of WAL, the present research addressed the role of agentic mechanisms to explain gender differences in leader emergence. Complementary to the meager literature on the agentic processes in leader emergence (e.g., Maurya and Agarwal, 2013; Elprana et al., 2015; Epitropaki, 2018), the present research found that women’s reluctance for leadership does not only come from being less motivated for leadership but also from perceived threat of leadership positions and accompanying emotion of worry about accepting such positions (Hoyt and Murphy, 2016; Alan et al., 2020).

Second, our findings contribute to the burgeoning attempts to expand the construct domain of leader emergence (cf., Hanna et al., 2021). Extant literature on leader emergence is relatively narrow in scope and focuses on who is “perceived as leader like” based on a person’s influence and dominance in informal group settings (Kaiser et al., 2008, p. 97). The current research addresses both opt-out and pushed-out processes (Kossek et al., 2017) operationalized as willingness for leadership and perceived leadership potential, respectively. Confirming the results of Aycan and Shelia (2019), we found evidence for the role of WAL in predicting both opt-out and pushed-out processes of leadership. As such, our research supports the notion that these two processes represent two intertwined, inseparable, and yet distinctive aspects of leader emergence. Following the example of the present research, we call for broadening the scope of contemporary and future leadership research to include possibilities of both self-selection and selection by others to formal leadership positions (cf. Aycan and Shelia, 2019) to provide comprehensive answers to the question of “how do leaders come about.”

Third, our findings have implications for the literature on stereotypes against women: (a) stereotype threat, and (b) stereotypical perception of women’s leadership potential. The finding that women with high WAL opt themselves out of leadership extends the stereotype threat literature in the domain of leadership (e.g., Hoyt and Murphy, 2016). WAL represents an anticipatory emotion that may be able to explain why situationally induced stereotype threat in a leadership context does not uniformly affect all women. We found that women with low WAL may be less susceptible to stereotype threat effects and, consequently, less likely to opt themselves out of leadership than women with high WAL. However, low (compared to high) WAL did not provide an advantage for women’s perceived leadership potential; women were pushed out of leadership regardless of their WAL levels. Our findings suggest that stereotypes against women are so pervasive that positive attributes, including low WAL and high competence, did not benefit women in their perceived leadership potential.

Finally, our findings also contribute to the meager literature on stereotypes about men in the leadership context. It appears that: (1) high WAL signals warmth for men, and (2) perception of warmth benefits men in receiving positive judgment of leadership potential. These findings support the growing literature on the role of communal qualities and androgyneity in leader effectiveness for males (e.g., Laustsen and Bor, 2017). Our findings imply that violating the stereotypical expectations (cf., EVT, Jussim et al., 1987) benefits men but not women in the context of WAL and leadership. In other words, men with high, compared to low, worries (which is against the stereotypical view of men in leadership, cf., Schein et al., 1996) received better ratings for their leadership potential, whereas women with low, compared to high, worries (which is against the stereotypical view of women, cf., Hoyt and Murphy, 2016) did not receive better ratings for their leadership potential.

Our findings are hoped to make contributions to practice. We attempted to offer a novel explanation for why women, including those with high potential, may choose to stay away from leadership positions. To empower more women and close the overall economic opportunity gap (World Economic Forum, 2018), organizations must not only create incentives to increase the attractiveness, aspiration, and motivation for leadership but also develop interventions that help to view the position of leadership as less threatening and worrisome, and thus address women’s WAL. Women may be informed about the finding that WAL is an ambivalent construct concerning leadership that is not necessarily obstructive to leadership; men’s WAL was unrelated to their willingness for leadership and even viewed as an advantage by others. Organizations may use this information to develop strategies that help women to overcome their worries about leadership or to reevaluate their worries in such a way that these worries do not turn into a self-set barrier to leadership. Information sessions explaining that women can be effective leaders, implementing organizational policies that allow for more flexible work schedules, and putting more women in charge to create positive role models may be ways of reducing women’s WAL (Olsson and Martiny, 2018). Additionally, intervention programs that make use of coaching, mentoring, emotion-regulation activities, or role modeling (see also, Martin et al., 2017) may help women to overcome their self-set barriers.

Our research further suggests that the perception of women as leaders is strongly driven by gender biases rather than by their qualifications. To alleviate the pushed-out effects on women’s leadership, interventions should also target those who are in charge of promotions in organizations. Raising awareness about gender-biased perceptions, adopting standard operations and practices that clearly define the criteria for promotion, and changing the organizational culture toward endorsing “atypical leaders” (Samdanis and Özbilgin, 2020) may help to promote a more gender-neutral and unbiased view on women’s leadership potential.

## Limitations and Future Research

Study 1 focused on the process of opting out of leadership using student samples who were charged with completing a risky decision-making task in a laboratory. One limitation here concerns the operationalization of leadership self-selection by using a single-item rating of willingness to decide on behalf of a group in Study 1. The possibility of discrepancy between intention and behavior has been discussed in the literature on attitudes (e.g., Ajzen et al., 2004). Our subjects may have not actually taken the leadership role in their group despite their stated willingness to do so. Yet, it should be noted that our probability measure of leadership was strongly tied to the actual behavior of becoming a leader (as the eventual “leader” was drawn among those who were willing to be the decision-makers). Moreover, the construct of interest – which is whether the participants are interested in making a decision on a specific task – seems suitable for a single-item assessment (for similar approaches, see Ertac and Gurdal, 2012; Born et al., 2020).

Studies 2 and 3 focused on being pushed out of leadership, where the participants were real-life supervisors who evaluated the leadership potential of real and imagined male and female subordinates. Even though external validity is increased by our use of students in an experimental setting and our use of supervisors in an organizational and experimental setting, the findings may fail to generalize to other leadership tasks (e.g., persuasion, negotiation, or conflict mediation), populations, and samples. Admittedly, the leadership-conducive effect of WAL among men may be context dependent and only advantageous in contexts where warmth is congruent with organizational goals (Eagly and Karau, 2002), which may have been the case for the retail organization from which data for Study 2 and Study 3 were collected. That is, warmth may fail to mediate WAL’s effect in other organizational contexts, or WAL may even exert a negative effect *via* decreased ratings of competence when the particular leadership situation requires to act more relentless. Thus, men with high WAL may have advantages in conflictual contexts that call for warm leaders who may be better able to smooth conflicts and promote cooperation.

This may also explain why the supervisors in Study 2 considered high WAL as an advantage for the male employees’ leadership potential. In their research, Gartzia and Van Knippenberg (2016) identified communion as a crucial feature of men’s leadership effectiveness. Communal traits among men engendered cooperative behavior, and this effect was especially pronounced in contexts that were dominated by men. Yet, it is equally possible that the stereotypical perception that men are competent (Cuddy et al., 2011) may have buffered the negative effect of WAL in Study 2, or that low competence of men was overlooked in favor of communal attributes, or that having worries was viewed as being overly ambitious. Thus, the leadership conducive effect of WAL among men may operate in a context-dependent manner, and be only advantageous where warmth is congruent with organizational goals (Eagly and Karau, 2002), or in conflictual contexts that call for warm and more “feminine” leaders who may be better able to smooth conflicts and promote cooperation (Tomlinson et al., 1997). The identification of possible boundary conditions to turn WAL into a leadership advantage requires further research in organizational settings where different styles of leadership are more desired.

In the future, researchers should consider the role of emotions, particularly WAL, and study how emotions shape the leadership processes of both women and men in conjuncture with different contexts where stereotypes against women are more versus less salient. Moreover, in order to identify the boundary conditions that prescribe whether the effect of WAL turns into an advantage or barrier, leadership research would benefit from a more systematic examination of the effects of WAL in organizational settings that involve different leadership requirements. Future research is also needed to understand how WAL is observable by others and how it affects others’ perceptions of leadership potential. Even though our research offers an initial insight, the issues of whether (and how) the behavioral reflection of WAL are different for men versus women, whether men and women are subject to biased evaluations despite equal reflections of WAL, or whether both the different reflections of WAL and the biased perceptions jointly affect men’s and women’s processes of being pushed out of leadership remain unresolved. Future research that compares self-reported WAL to other-assessments of WAL by also assessing the physiological and behavioral manifestations of WAL may help to find a remedy.

## Conclusion

In three studies using experimental and field study methods, we examined the role of WAL for men and women in opting out and being pushed out of leadership. While the WAL of women operated as a self-set barrier in terms of their willingness for leadership (i.e., opt-out), men with high WAL did not abstain from assuming leadership. Moreover, high WAL even turned into a leadership advantage among men by enhancing their perceptions of leadership potential (i.e., pushed out), most likely *via* enhanced perceptions of warmth. When judging women’s leadership potential, however, their WAL seems to be irrelevant, suggesting that women’s leadership potential may be evaluated in light of the gender stereotypes. As such, while WAL seems to represent an influential construct to predict leadership opt-out processes of women, it turned out to be irrelevant for predicting women’s pushed-out processes. Yet, further research is needed to examine how WAL would operate on women to be pushed out of leadership in work settings that are more or less afflicted with gender biases and stereotypes.

## Data Availability Statement

The raw data supporting the conclusions of this article will be made available by the authors, without undue reservation.

## Ethics Statement

The studies involving human participants were reviewed and approved by the Institutional Review Board of Koç University (Turkey). The patients/participants provided their written informed consent to participate in this study. Written informed consent was obtained from the individual(s) for the publication of any potentially identifiable images or data included in this article.

## Author Contributions

AK, AB, and ZA involved in planning and designing the research and formulated the research questions and hypotheses for all three studies included in the manuscript. AK and AB prepared all data collection material and were actively involved in collecting the research data. AK performed the data analysis for Study 1 and Study 2. GK performed the data analysis for Study 2. All authors actively contributed to writing and editing parts of the manuscript.

## Conflict of Interest

The authors declare that the research was conducted in the absence of any commercial or financial relationships that could be construed as a potential conflict of interest. ZA is one of the co-authors of this manuscript and also one of the editors of the Special Issue Topic.

## Publisher’s Note

All claims expressed in this article are solely those of the authors and do not necessarily represent those of their affiliated organizations, or those of the publisher, the editors and the reviewers. Any product that may be evaluated in this article, or claim that may be made by its manufacturer, is not guaranteed or endorsed by the publisher.

## Footnotes

1 The participants in Study 1 and Study 2 and 3 do not necessarily represent the values of the typical Turkish culture. The private university whose students participated in Study 1 is a world-ranked research university with an American education system. The company whose supervisors and employees participated in Studies 2 and 3 is a multinational corporation with a strong Western organizational culture.

2 All 71 groups consisted of five members. However, when participants did not show up to their laboratory session, they were replaced by confederates who acted as participants.

3 We are aware that leadership, in practice, describes a multi-faceted concept that extends beyond being willing to be a group’s decision-maker for a single risk-involving task. However, readiness for making risky decisions represents a core component of executive decision-making and leadership (see also Ertac and Gurdal, 2012).
